# A New Theory of Gender Dysphoria Incorporating the Distress, Social Behavioral, and Body-Ownership Networks

**DOI:** 10.1523/ENEURO.0183-19.2019

**Published:** 2019-12-11

**Authors:** Stephen V. Gliske

**Affiliations:** Department of Neurology, University of Michigan, Ann Arbor, Michigan 48109

**Keywords:** body-ownership network, distress, gender dysphoria, sensory perception, social behavioral network, transgender

## Abstract

When postmortem studies related to transgender individuals were first published, little was known about the function of the various identified nuclei. Now, over 2 decades later, significant progress has been made associating function with specific brain regions, as well as in identifying networks associated with groups of behaviors. However, much of this progress has not been integrated into the general conceptualization of gender dysphoria in humans. I hypothesize that in individuals with gender dysphoria, the aspects of chronic distress, gender atypical behavior, and incongruence between perception of gender identity and external primary sex characteristics are all directly related to functional differences in associated brain networks. I evaluated previously published neuroscience data related to these aspects and the associated functional networks, along with other relevant information. I find that the brain networks that give individuals their ownership of body parts, that influence gender typical behavior, and that are involved in chronic distress are different in individuals with and without gender dysphoria, leading to a new theory—that gender dysphoria is a sensory perception condition, an alteration in the sense of gender influenced by the reflexive behavioral responses associated with each of these networks. This theory builds upon previous work that supports the relevance of the body-ownership network and that questions the relevance of cerebral sexual dimorphism in regard to gender dysphoria. However, my theory uses a hierarchical executive function model to incorporate multiple reflexive factors (body ownership, gender typical/atypical behavior, and chronic distress) with the cognitive, reflective process of gender identity.

## Abstract (precis)

When postmortem studies related to transgender individuals were first published, little was known about the function of the various identified nuclei. Now, over 2 decades later, significant progress has been made associating function with specific brain regions, as well as in identifying networks associated with groups of behaviors. However, much of this progress has not been integrated into the general conceptualization of gender dysphoria in humans.

## Significance Statement

My new model highlights connections between multiple dimensions of gender dysphoria and behavioral neuroscience data, explaining the experience of gender dysphoria using relevant neural substrates and networks. This biology/symptom-based approach provides an updated theory of gender dysphoria, fostering new hypotheses to advance basic understanding of the condition. If supported by future studies, this theory could be the next step towards discovering currently unseen doors for improving the lives of those with gender dysphoria.

## Introduction

Just over 20 years ago, a publication reported the first observed neurobiological difference between cisgender and transgender individuals (Zhou et al., 1995). In particular, the bed nucleus of the stria terminalis (BNST) was found to have a smaller average size in male-to-female (MtF) transgender individuals, with a size more similar to that of an average cisgender female than cisgender male. For context, see the accompanying commentary (Breedlove, 1995). More succinctly, Breedlove was described in a *New York Times* article as expressing that the “function of the bed nucleus in human behavior, sexual or otherwise, remained ‘a complete black box’” (Angier, 1995). Interpretation of the BNST results at that time thus focused on the size difference rather than the function. As MtF transgender individuals had a size more similar to their desired gender than assigned gender, these data supported the theory that distress in gender dysphoria was due to an anatomic incongruence between brain and body sex. The incongruence was then specifically stated to be that transgender individuals have brain sex opposite to their gender assigned at birth. For clarity, I will refer to this theory as the opposite brain sex theory, which is in the category of theories involving atypical cerebral sexual differentiation.

Today, the BNST is no longer a black box but has several identified functions. For example, the BNST is a key component of the fear/distress network (Lebow and Chen, 2016; Tillman et al., 2018). Although chronic distress is a defining characteristic of gender dysphoria, the connection between the functional role of the BNST and its association with gender dysphoria appears to have received little consideration. In contrast, the connection between anatomic changes in the body ownership network and gender dysphoria has been a focus of several recent studies (Burke et al., 2017; Manzouri et al., 2017; Manzouri and Savic, 2019). The results on both the distress and body ownership networks suggest a theory in which each aspect of gender dysphoria is explained by the functional significance of known neuroanatomical differences. Specifically, I hypothesized that in individuals with gender dysphoria, the aspects of chronic distress, gender atypical behavior, and incongruence between perception of gender identity and body sex are all directly related to the functional implications of the underlying differences in neurobiology. I considered the plausibility of this hypothesis by examining published literature regarding the function and behavioral roles of neuronal substrates found to be different in transgender individuals.

After considering this hypothesis, I present a new theory of gender dysphoria, consistent with the latest neuroscience data, that stands in contrast to the common opposite brain sex theory and builds on the work relating body perception with gender dysphoria (Burke et al., 2017; Manzouri et al., 2017; Manzouri and Savic, 2019). I denote this new theory as the multisense theory of gender dysphoria. This new theory focuses on function, including sense of gender and its inputs, rather than male/female dichotomy in anatomic size and shape (the focus of the opposite brain sex theory). For clarity, in this document I use “sense of gender” to refer to the emergent sense arising from the function of multiple networks, and “brain sex” to refer to anatomic characteristics of the brain relative to male/female dichotomy. I also use the term “transgender” throughout this manuscript, though I recognize that some references instead use the word transsexual to refer to the same concept. I observe, based on previously published data, that the primary mechanism behind the experience of gender dysphoria appears not to be that the anatomic brain sex is opposite to gender assigned at birth. Instead, I propose that systemic changes in functional networks, specifically the distress, social behavioral, and body-ownership networks, result in the incongruence between sense of gender and gender assigned at birth.

## Background material

The new theory is rooted in published neuroscience data related to gender dysphoria and behavioral roles of the associated neuronal substrates. Most of this information has become available within the last 20 years, with more than half of the cited references being published within the last 6 years. I organized available information around three key dimensions of gender dysphoria, consistent with the Diagnostic and Statistical Manual of Mental Disorders, version 5 (DSM-V). Specifically, the three dimensions were (1) chronic distress, (2) gender nonconformity, and (3) incongruence between perception of gender identity and body sex. In this categorization, the desire to become a gender other than assigned gender is viewed as a resultant effect of these three dimensions. The presence of dimensions 2 and/or 3, without severe distress (dimension 1), does not constitute gender dysphoria according to the DSM-V.

### Dimension 1: chronic distress

The key neuronal substrate for processing distress is the central extended amygdala, which includes the BNST and central medial amygdala. The extended amygdala is implicated in psychiatric conditions including extended duration fear states such as chronic dysphoria (Lebow and Chen, 2016). The BNST is also a component of several important networks, including the social behavioral network (Newman, 1999), the mesolimbic reward system (O’Connell and Hofmann, 2011), the hypothalamic–pituitary–adrenal axis (related to acute stress; Zhu et al., 2014), and the sleep/wake system (Saper et al., 2005a,b). Altered size of the BNST was the first noted anatomic change associated within MtF transgender individuals (Zhou et al., 1995). The BNST is also part of a larger distress-processing network, involving the periaqueductal gray, anterior insula, dorsolateral prefrontal cortex, mid-cingulate cortex, and orbitofrontal cortex (Tillman et al., 2018). Two additional nodes of the distress network, the anterior insula and orbitofrontal cortex, have also been found to be altered in transgender individuals (Zubiaurre-Elorza et al., 2013; Manzouri et al., 2017; Fig. 1).

**Figure 1.** Networks related to key dimensions of gender dysphoria. Each box represents nuclei or brain regions involved in these networks. Red asterisks are included in boxes where the following regions/nuclei have known anatomic changes associated with transgender individuals (Smith et al., 2015; Guillamon et al., 2016; Altinay and Anand, 2019): anterior hypothalamus (AH; Garcia-Falgueras and Swaab, 2008); BNST (Zhou et al., 1995); anterior insula (aINS) and orbitofrontal cortex (OFC; Zubiaurre-Elorza et al., 2013); superior parietal lobe (SPL; Lin et al., 2014); and intraparietal sulcus (IPS; Case et al., 2017). Connections are based on the studies by Kong et al. (2010), Newman (1999), and Tillman et al. (2018). AH, Anterior hypothalamus; cAMY, central amygdala; DLPF, dorsolateral prefrontal cortex; LS, lateral septum; MCC, mid-cingulate cortex; mPOA, medial preoptic area; PAG, periaqueductal gray; Teg, tegmentum; VPM, ventral premotor cortex. Solid lines with arrows represent anatomical connections, while dash-dotted lines represent known functional connections.

### Dimension 2: gender nonconformity

Most behaviors associated with being typical of a given gender are under control of the social behavioral network. Categories of behaviors typically associated with this network include parental, sexual, and aggressive behaviors (Newman, 1999). The social behavioral network is applicable for many mammalian species (Goodson and Kingsbury, 2013). While the basic understanding of the network is based on animal studies, the results are thought to generalize well across mammalian species, including humans, at least to the extent that these regions are involved in the same category of behaviors (Goodson and Kingsbury, 2013; Kelly and Goodson, 2014; Johnson and Young, 2017). In animal models, the types of behaviors related to this network also appear similar in both sexes (Goodson and Kingsbury, 2013), though the actual behaviors are gender specific. For example, typical male and female parental roles are not identical, though the social behavioral network does relate to parenting roles in both sexes. The social behavioral network is commonly listed to contain the medial extended amygdala (including the BNST and central medial amygdala), the lateral septum, the medial preoptic area, the anterior hypothalamus, the ventromedial hypothalamus (VMH), ventrolateral hypothalamus, paraventricular nucleus of the hypothalamus, and two midbrain structures, the tegmentum and periaqueductal gray (Newman, 1999; Goodson and Kingsbury, 2013; Kelly and Goodson, 2014; Fig. 1). Postmortem studies identified the following two regions of the social behavioral network being altered in MtF transgender individuals: the third interstitial nucleus of the hypothalamus (INAH3), part of the anterior hypothalamus, and the BNST (Zhou et al., 1995; Garcia-Falgueras and Swaab, 2008).

### Dimension 3: incongruence and body ownership

The involvement of the body-ownership network (Tsakiris, 2010) in gender dysphoria can best be described by first considering how this network is studied in other contexts. The network has often been examined using the rubber hand illusion, whereby an individual is made to feel ownership over a rubber hand by time-locked visual and tactile stimulation to both the observed rubber hand and the unobserved real hand. Time-locked visual and tactile stimulation have also been used to create the illusion of ownership of an entire body that is not one’s own. The illusion even persists if the individual shakes hands with what looks like their actual body (Petkova and Ehrsson, 2008). The illusion involves subconscious processing, which is closely connected with other systems. For example, causing one to feel ownership of a more obese body can cause activation of the distress network, particularly the insula and anterior cingulate cortex (Preston and Ehrsson, 2016), whereas the illusion of being invisible can reduce subjective and objective social stress measures (Guterstam et al., 2015). Ownership of an artificial limb has also been induced in amputees by replacing the tactile stimulus with electrical stimulation (Collins et al., 2017). The body-ownership network is considered (Grivaz et al., 2017) to include the insula (particularly the left anterior insula), the right ventral premotor cortex, and portions of the posterior parietal cortex (specifically the right and left intraparietal sulci and left superior parietal lobule; see also discussion in Manzouri et al., 2017; Fig. 1).

The literature based on human data, which connects gender dysphoria with the body-ownership network and body perception, has been continually growing over the last decade. Some early work identified the involvement of the cingulate and insula but failed to associate them with their roles in body perception or distress (Nawata et al., 2010; Zubiaurre-Elorza et al., 2013), having their interpretation instead focused on cerebral dimorphism. Savic and Arver (2011) recognized the involvement of body perception networks in gender dysphoria as early as 2011 and have since published a stream of articles further reinforcing its relevance. Some studies focused purely on anatomic measurements (Burke et al., 2017; Manzouri et al., 2017; Manzouri and Savic, 2019). Other studies used images of the bodies of research subjects morphed to look more like the opposite gender (Feusner et al., 2016, 2017; Burke et al., 2019). Hormonal treatments were found to reverse the observed anatomic effects and increase consistency between self-perception and actual body image (Burke et al., 2018; Kilpatrick et al., 2019). The effect of sexual orientation was also found to be a major confounding factor, in that some changes in earlier work thought to be associated with gender dysphoria were found to be explained better by the sexual orientation of the subjects (Burke et al., 2017; Manzouri and Savic, 2019). However, regions of the body-ownership network remained significant even after controlling for sexual orientation (Burke et al., 2017; Manzouri and Savic, 2019). Note that homosexual is defined in these studies relative to gender assigned at birth (e.g., an androphylic MtF transgender individual would be labeled as homosexual). One of the regions identified in these studies (Nawata et al., 2010; Zubiaurre-Elorza et al., 2013; Manzouri et al., 2017), the anterior insula, is a common node in both the distress and body-ownership networks, and is interconnected with the central extended amygdala and periaqueductal gray (Kong et al., 2010; Tillman et al., 2018). Beyond the work of Savic (Feusner et al., 2016, 2017; Burke et al., 2017, 2018, 2019; Manzouri et al., 2017; Manzouri and Savic, 2019; Kilpatrick et al., 2019), results from a task-based study focused on the body representation network in transgender individuals, which included changes in the postcentral gyrus and superior parietal lobule (Lin et al., 2014). Lin et al. (2014) motivated that study by claiming that the involvement of the body-ownership network is a consequence of “dissonance between their biological sex and gender identity.” However, all available relevant data are correlational and do not constrain whether changes in body ownership cause, or are caused by, the perception of dissonance.

The body-ownership illusion studies demonstrated that the visual and tactile stimulation must be time locked to lead to a sense of body ownership, suggesting that interference in the normal processing of this stimulation could lead to a loss of body ownership. For example, xenomelia is a condition in which individuals feel a given body part is not their own, feel distress, and desire to have it removed. Changes have been observed in the body-ownership network using MRI data (Hilti et al., 2013) and cellular activation measured by MEG (McGeoch et al., 2011). Similar changes in MEG activation have been observed in transgender individuals. For example, Case et al. (2017) recorded MEG from female-to-male (FtM) transgender individuals and controls during tactile stimulation to breast and hand. In the FtM transgender individuals, the evoked potential response from breast stimulation was reduced relative to hand stimulation, particularly in the intraparietal sulcus (part of the body-ownership network) and primary motor and somatosensory cortices. Additional electrophysiology results are discussed by Smith et al. (2015). Thus, sensory perception related to body ownership and both gray and white matter in the body-ownership network (particularly the anterior insula, intraparietal sulcus, and superior parietal lobule) are directly linked with transgender individuals (Fig. 1, asterisks).

### Additional relevant data

I next list additional information about gender dysphoria, which should be considered when evaluating hypotheses regarding its cause. Gender dysphoria is a separate construct than just being gender atypical (American Psychiatric Association, 2013), and gender-atypical individuals do not necessarily experience significant distress or a decreased ownership of their assigned gender. Additionally, gender dysphoria in younger children has been shown to resolve before puberty without treatment—with some estimates of a resolution rate between 55% and 80% (Drummond et al., 2008; Steensma et al., 2011). Common conditions comorbid with gender dysphoria include autism (Strang et al., 2018) as well as other factors typically ascribed to psychosocial factors, specifically anxiety, depression, suicidal ideation, and suicide. Treatment for gender dysphoria currently involves gender reassignment, which can include changing one’s social presentation and identification as well as bodily alteration via hormonal therapy and/or surgery. Treatments are successful at accomplishing the gender reassignment (for review, see World Professional Association for Transgender Health, 2011; Hembree et al., 2017), but outcome measures directly related to distress or body ownership have not typically been considered or reported in the past. However, two recent publications did consider perception of body ownership, but did not specifically consider distress. They found that hormones reverse the anatomic changes in the body-ownership network and increase own-body self-congruent rates (Burke et al., 2018; Kilpatrick et al., 2019). The exact cause of gender dysphoria is unknown, but the cause is believed to be biological in nature.

### Synthesis of existing data

Previously published data support my hypothesized direct connection among the three specified dimensions of gender dysphoria and the functional roles of the implicated neuronal substrates and networks. Chronic distress is a defining characteristic of gender dysphoria, and multiple nodes of the distress processing network have been found to be altered in transgender individuals using multiple measurement modalities. Behavior atypical of assigned gender is common in individuals with gender dysphoria (with some exceptions depending on age of onset and sexual orientation), and two nodes of the social behavioral network (the network involved in gender-typical behavior) have been found to be different in transgender individuals. Last, the network for body ownership and self-perception have also been found to be altered, showing changes in white matter, gray matter, functional connectivity, and response to stimuli, including altered sensory response from body parts perceived as incongruous with desired identity. Correlations were also found between affirming hormonal treatment and changes in anatomy of the body-ownership network. Thus, the distress, social behavioral, and body-ownership networks each directly match a key dimension of gender dysphoria, and each network has multiple nodes observed to be altered in transgender individuals (Fig. 1).

Published data do not sufficiently address causality between gender dysphoria and alteration in these three networks. It is possible that the changes in all of these networks are secondary to gender dysphoria, a concept claimed in previous literature for the body-ownership network (Lin et al., 2014). However, the data also allow the following alternate interpretation: that changes in these networks are causal to the experience of chronic distress, gender atypical behavior, and incongruence between perceived gender identity and assigned gender. This view does not minimize the known negative impact of various external factors but instead focuses on developing an understanding of what gender dysphoria actually is at a biological level.

## The new multisense theory of gender dysphoria

In contrast to existing theories of gender dysphoria, I propose a new theory (the multisense theory) wherein alteration (possibly activational or organizational) in the interacting distress, social behavioral, and body-ownership networks leads to dynamic changes in network activity, causing the subjective experience of gender dysphoria and possible additional, concomitant, observable anatomic changes. While a variety of neuroanatomical changes have been noted (for review, see Smith et al., 2015; Guillamon et al., 2016; Altinay and Anand, 2019), my view specifically addresses the functional significance of the observed changes in the distress network, social behavioral network, and body-ownership network, including the neuronal substrates of the BNST, anterior hypothalamus (encompassing the INAH3), anterior insula, intraparietal sulcus, superior parietal lobule, and orbitofrontal cortex. Changes in these substrates support my hypothesis that, in individuals with gender dysphoria, the aspects of chronic distress, gender-nonconforming behavior, and incongruence between perception of gender identity and body sex are all directly related to the underlying differences in neurobiology.

I also model that senses based on these networks are integrated with each other and other factors, resulting in an overall sense of gender (Fig. 2). The underlying neurobiology would influence how much an individual feels chronic distress, how much they desire to act in a manner consistent with their gender role, and how much they feel the gendered aspects of their body belong to them—all of which then contributes to the extent to which an individual feels that their gender matches that which was assigned at birth (i.e., their overall sense of gender). While the experimental evidence is strongest for the body-ownership/perception network and weakest for the social/behavioral network, I allow that the relative weight and causal order of these factors may be different in different individuals. External factors can also influence the sense of gender either directly or via affecting the reflexive senses of distress or behavior relative to gender roles. While there are insufficient data to understand the impact of the changes in the precuneus (Manzouri and Savic, 2019), a region that integrates sensory information, a key component of my theory is the integration of multiple senses and factors to form an overall sense of gender.

**Figure 2.** Diagram of the multisense theory of gender dysphoria. The overall sense of gender in an individual is modeled as a neurobiological, reflective sense, integrating information from multiple senses and stimuli (bold arrows). This sense of gender is framed relative to gender assigned at birth (e.g., am I the gender that was assigned at birth?) rather than an absolute male/female dichotomy (e.g., am I female?). Each of the three listed reflexive senses (purple boxes) relate to a specific dimension of diagnostic criteria for gender dysphoria as well as a matching functional network with nodes known to be altered in transgender individuals (Fig 1). The interaction between sense of gender and these three reflexive senses may be bidirectional. External factors (green boxes) influence sense of gender either directly (bold arrow) or indirectly via affecting the reflexive senses. The model can also be extended to include additional internal and external factors. The diagram represents a dynamic network, not a specific causal pathway, and includes potentially complex interactions and feedback loops.

## Discussion

### Consistency of the new theory with existing data

#### Dynamic activity on functional networks

The multisense theory proposes that gender dysphoria is not merely due to static changes in anatomy, as in the previous opposite brain sex theory, but instead includes dynamic activity on interacting, functional networks. This dynamic aspect can explain the distinctness of gender dysphoria from being gender atypical, accounts for the variety of onset ages and both persistent and desistant cases, and is still consistent with the anatomic findings. Changes in sex hormones due to puberty (or aging) could also affect these identified networks, explaining both resolution without treatment in childhood-onset cases and the possibility of late-onset cases. Data now support that each of these dimensions (distress, gender conformity, and body ownership/perception) are associated with specific functional neural networks, which is part of the basis of the multisense theory. The multisense theory is also consistent with recent meta-analyses (Smith et al., 2015; Guillamon et al., 2016; Altinay and Anand, 2019), as follows: the data presented show that the brains of transgender individuals are not simply altered along a male/female dimension to be more like their desired gender, even in studies that controlled for sexual orientation. Thus, overall, the available published data are consistent with the multisense theory of gender dysphoria.

#### Comorbid conditions

The comorbid conditions of anxiety, depression, suicidal ideation, and suicide are commonly attributed to having the opposite brain sex as gender assigned at birth as well as psychosocial factors. The latest data challenge that view regarding anatomic brain sex and suggest that altered neuroactivity in the identified networks could also play a key role in these comorbidities. In particular, the distress network, especially the BNST, extended amygdala (Lebow and Chen, 2016), and potentially the insula (Carlson et al., 2011; Tillman et al., 2018), are involved in mood regulation conditions, such as anxiety and depression. Another region altered in individuals with gender dysphoria, the anterior cingulate, is strongly associated with depression (Drevets et al., 2008; Bunney et al., 2015). Recent data also suggest that self-perception, related to the body-ownership network, is altered in individuals with autism (Ropar et al., 2018), another known comorbidity of gender dysphoria. Thus, the underlying mechanisms causing gender dysphoria may also be directly contributing to comorbid conditions, in addition to the indirect contribution mediated by external factors.

### Comparison with other theories of gender dysphoria

A prevalent and early theory of gender dysphoria is that it is a manifestation of an actual difference between the person and gendered aspects of their body, assuming that the individual’s sense of body ownership and gender identity (their subjective experience) is fully correct (Gooren, 2006). This theory is one basis for sex reassignment as a therapy for gender dysphoria (Fisk, 1974). The initial neuroanatomical studies, which first became available in 1995, also supported this view (Zhou et al., 1995; Garcia-Falgueras and Swaab, 2008). In these studies, an anatomic difference was found in a sexually dimorphic brain area, with the transgender individual’s measurements being closer to that of their desired gender rather than their gender assigned at birth. The associated distress was attributed to the incongruence and/or psychosocial and cultural factors. Gradually, it became clear that both structural and functional networks were likely involved (Garcia-Falgueras and Swaab, 2008). However, only recently have data begun to be available regarding the biological basis of self-identity and body ownership and its connection with gender dysphoria (Burke et al., 2017; Case et al., 2017).

Another modification was needed when *in vivo* imaging data later demonstrated that brains of transgender individuals also have unique differences relative to cisgender individuals that are not fully explained by altered cerebral sexual differentiation, even when controlling for sexual orientation (for papers reviewed, see Smith et al., 2015; Guillamon et al., 2016). One suggestion was that incongruence in limited brain regions is sufficient to cause gender dysphoria (Guillamon et al., 2016). However, anatomic brain sex only appears to be distinctive at the whole-brain level, rather than at the level of individual nuclei, within individuals without gender dysphoria (Chekroud et al., 2016; Rosenblatt, 2016). Thus, anatomic incongruence (i.e., having a size/shape more like the opposite gender) in limited regions is typical in individuals without gender dysphoria and is not likely to be sufficient to cause gender dysphoria.

The multisense theory, however, does not preclude that some anatomical changes associated with gender dysphoria may appear as atypical cerebral sexual dimorphism nor does it preclude involvement of sex hormones; the multisense theory interprets these changes based on the functional implications. For example, the functional significance of alteration in the BNST (Zhou et al., 1995) was not understood until long after 1995, and thus these results were originally interpreted relative to sexual dimorphism. Similarly, the functional significance of some other alterations is not yet fully understood. If such alterations are fundamental to gender dysphoria and not just secondary effects, then the prediction of the multisense theory is that the functional significance will relate to the distress, body-ownership, and/or social behavioral network, with the level of sexual dimorphism being less relevant.

Another modification to the opposite brain sex theory was recently proposed by Altinay and Anand (2019). In this theory, the sense of gender does not arise from limited cerebral sexual dimorphism, but rather from “brain gender,” which they defined as “gender identity specific brain architecture and organization.” While Altinay and Anand (2019) suggest that brain gender might be the body ownership network, they do not clearly define what brain gender actual means in terms of neurobiology, and instead focus on interactions with external stimuli and how this would feed into distress via cognitive dissonance. The multisense theory also recognizes the influence of external stimuli (Fig. 2), including how cognitive dissonance could increase distress. However, the multisense theory does not encapsulate all anatomic changes into a brain gender or place distress as only secondary to other changes. Instead, the multisense theory details how changes in specific networks relate to specific reflexive senses (which would impact the overall sense of gender) and allows for the possibility that several of these networks could be causal to the condition in some individuals.

One other theory of gender dysphoria has also been proposed that does not directly involve alterations in cerebral sexual differentiation. Manzouri and Savic (2019) “suggest that [gender dysphoria] is… specifically linked to cerebral networks mediating self-body perception” rather than a “less pronounced cerebral sex dimorphism,” an idea expressed in multiple articles from their group. The multisense theory includes this concept as one component but also extends beyond this idea to explain other symptoms of gender dysphoria by incorporating other important networks.

One might argue that the general success of gender identity affirmation treatments for gender dysphoria supports only theories based on a brain/body sex incongruence. However, the argument depends on the mechanisms of how treatments affect symptoms, which is currently unknown. Both males and female brains need estrogen and testosterone. Changes in these hormones could potentially affect the body-ownership, social behavioral, and/or distress networks. For example, the impact of affirming hormone treatment (testosterone for FtM individuals, estrogens, and anti-androgens for MtF individuals) was recently studied for individuals with gender dysphoria. In both FtM and MtF individuals, hormone treatment increased own-body self-congruence rates (although no surgical alterations were yet performed), and it also resulted in cortical thickness returning to be more like that of individuals without gender dysphoria (Kilpatrick, et al., 2019). The exact mechanism is unknown, but both hormone treatments would increase estrogen in the brain, either directly (MtF) or indirectly via aromatization (FtM). Thus, the partial efficacy of current treatments may be due, in part, to the hormones indirectly influencing the body-ownership, distress, and/or social behavioral networks. Additionally, external factors such as diagnosis with gender dysphoria or receipt of a treatment plan could also impact the sense of gender and symptoms of gender dysphoria, including potentially increasing or decreasing distress. Given that the mechanism leading to the efficacy of current treatments is not yet well understood, the efficacy of current treatment thus does not exclude the multisense theory of gender dysphoria and provides little disambiguation between theories of gender dysphoria.

### Interaction with other networks

#### Sexual and romantic partner preference

Subtypes of gender dysphoria have been proposed based on sexual orientation and onset age (Blanchard, 1989), though the subtype labels do not necessarily match the subjective experience of individuals with gender dysphoria (Gooren, 2006). Another recent article concluded that MtF individuals with early- and late-onset gender dysphoria have statistically significant differences in their sexual orientation, though the data show a variety of sexual orientations being present in both subtypes (with early-onset cases being only 52.6% attracted to men; Zavlin et al., 2019). The multisense theory allows for two possible explanations for correlation between onset age and partner preference among individuals with gender dysphoria, which are detailed in the next two paragraphs. These two possibilities are not mutually exclusive.

The first explanation is that gender dysphoria and partner preference represent different underlying mechanisms, but interaction between the mechanisms causes the appearance of subtypes. While gender dysphoria appears related to internally focused senses (sense of own gender, described earlier), partner preference appears to be related to externally focused senses, particularly a sense of the gender of others. For example, a recent MRI study suggested that homosexuality may involve altered interpretation of external sensory stimuli (Manzouri and Savic, 2018), which is consistent with earlier work from their group regarding the processing of smell and partner preference (Savic et al., 2005; Berglund et al., 2006). Given the available data, detailed below, I hypothesize that partner preference is connected with the neurohormone vasopressin in brain regions related to social recognition (specifically, the lateral septum), affecting the subconscious, sensory response to the gender of others. In some cases, this change could result in an equivalent subconscious response to all genders (bisexual partner preference). In other cases, this change, combined with other factors, could cause the perception that the opposite gender is too different to be a sufficiently compatible partner (homosexual partner preference). Human data supporting this hypothesis include the study by Swaab and Hofman (1990), which found that the number of vasopressin-secreting neurons in the suprachiasmatic nuclei (SCNs) of homosexual males were on average three times larger than that in male and female heterosexual controls. At the time, interpretation focused on the overall shape (homosexual males having an overall shape more like females than males), rather than the number of vasopressin-secreting cells in homosexual men being distinct from both male and female heterosexual individuals. In animals, increases in the number of vasopressin-secreting neurons and bisexual and homosexual behavior were also observed in male rats treated with an aromatase inhibitor during the perinatal SCN developmental period (Bakker et al., 1993; Swaab et al., 1995). Aromatase enzyme knock-out (ArKO) male mice exhibited decreased social recognition (vocalizing toward both genders instead of just females), decreased habituation to test female mice, and decreased vasopressin levels in the lateral septum (a node in the social behavioral network); the behavior and vasopressin levels in the lateral septum were restored to control levels with adulthood administration of dihydrotestosterone and estrogen (Pierman et al., 2008). Other rat studies also support vasopressin in the lateral septum having a role in social recognition (Bychowski et al., 2013). Human studies corroborate these findings, with data supporting the role of vasopressin in bonding (Atzil et al., 2012), cooperative risk (Brunnlieb et al., 2016), and other aspects of social recognition and behavior (for review, see Johnson and Young, 2017). In humans, it is possible that an increased number of vasopressin-secreting cells in the SCN, as found in homosexual men, could lead to too low of levels of vasopressin in the lateral septum due to compensatory effects. Changes in septal areas have actually been associated with partner preference in humans (Poeppl et al., 2016). Thus, while more research is needed in humans (especially females) to develop a complete model of partner preference and its relationship to gender dysphoria, the data suggest the plausibility of my hypothesis regarding partner preference, vasopressin, and the lateral septum. Interaction among these closely connected regions could thus explain the subtypes, though stronger data are needed before including these factors in my multisense model of gender dysphoria. Evidence does suggest that partner preference, like gender dysphoria, also involves sensory perception.

The second explanation for the correlation between onset age and partner preference among individuals with gender dysphoria centers on relative timing. Assume that partner preference is encoded in the brain in the relative terms of “same” and “different” (as sense of gender is encoded in the brain in the multisense theory) rather than absolute “male” and “female.” Then an individual attracted to the opposite gender could be attracted to either males or females depending on what they sensed their gender to be when they developed partner preference; likewise, individuals attracted to the same gender could also be attracted to either males or females. Late-onset cases are likely to occur after the development of partner preference. Thus, the following subtypes emerge: individuals with early-onset gender dysphoria would tend to be labeled by Blanchard (1989) as a homosexual subtype, and most individuals with late-onset gender dysphoria would be labeled by Blanchard (1989) as a nonhomosexual subtype. It is not yet clear why the subtypes appear stronger in males than females. However, the defining characteristic of the subtypes appears to be the onset age of gender dysphoria, not the sexual orientation.

#### Sleep/wake and circadian

Each of the three identified networks has significant overlap and anatomic connections with the sleep/wake and circadian-timing systems. This includes the VMH (social behavioral network; Orozco-Solis et al., 2015, 2016), the BNST (distress and the social behavioral network), lateral septum (social behavioral network; Saper et al., 2005b), and the insula (distress and body ownership networks; Chen et al., 2016). Circadian dysregulation may also be involved in the association between gender dysphoria and its comorbidities. For example, circadian dysregulation in the anterior cingulate, a region found to be different in individuals with gender dysphoria, is associated with depression (Bunney et al., 2015). Genetic studies also provide weak support for a connection between gender dysphoria and sleep/circadian regulation, though the data are not overly specific. While results from large-scale genetic association studies are not yet available, the candidate genes identified in small cohort studies are all associated with sex hormones (Henningsson et al., 2005; Hare et al., 2009; Ujike et al., 2009; Fernández et al., 2014a,b; Cortés-Cortés et al., 2017) or the ryanodine type-3 receptor (Yang et al., 2017), all of which influence the sleep/wake and circadian systems (Vasalou and Henson, 2010; Whitt et al., 2018). Thus, in general, the available data support possible relationships between sleep/circadian regulation and gender dysphoria, though the data are not definitive and do not quantify the relative importance of sleep/circadian factors. I do note that one case study makes an unsupported statement that sleep disorders are higher in children with gender dysphoria (Kern et al., 2014), though direct empirical evidence does not seem to be available. Thus, there is need for future studies to understand how sleep/circadian regulation influences gender dysphoria and its comorbidities, how treatments for gender dysphoria influence sleep via sex hormone changes, and the extent to which sleep disorders are comorbidities of gender dysphoria.

### Future directions

The multisense theory of gender dysphoria suggests future research studies that could improve the understanding of gender dysphoria and provide data to further test/validate related theories. One direction of future research would be to continue to disentangle the association of neural substrates and networks with each of the three noted dimensions of gender dysphoria. Additional controls are needed, such as individuals with gender-atypical behavior during childhood or other ages without gender dysphoria but of each sexual orientation, and individuals with other chronic distress or body-ownership conditions, such as body dysmorphic disorder, xenomelia, anorexia, and depersonalization. This will allow further stratification of the relationship between behavioral effects and specific neural networks. Additionally, it will be essential to assess individuals with gender dysphoria rather than the larger population of transgender individuals, an important distinction that is present in some recent work (Feusner et al., 2017). Not all transgender individuals necessarily have gender dysphoria.

Future studies should also address how treatment affects specific dimensions of gender dysphoria, which is quite limited in current data. Treatment outcome measures have often been designed to assess satisfaction with new gender and the effectiveness of the gender reassignment (World Professional Association for Transgender Health, 2011; Hembree et al., 2017). These measures do not adequately assess the dimension of distress, the effect on body ownership, or the impact of hormonal treatments on sleep and circadian function. For example, recent data suggest that hormone treatment alone may directly address some of the underlying neurobiology and reduce the incongruence of own-body perception (Kilpatrick et al., 2019). I additionally recommend that future research regarding treatment outcomes specifically and directly assess distress and body ownership in their primary outcomes, as well as the effects on sleep/wake and circadian phases in their secondary outcomes.

The multisense theory can also help to facilitate future research separating out predisposing, precipitating, and perpetuating factors of gender dysphoria. For example, an increase of distress, due to internal or external factors could potentially cause an atypical child with a predisposition for gender dysphoria to develop the condition, or, alternately, cause an individual to have persistent gender dysphoria when it otherwise would have resolved. Extending the framework of the multisense theory to include predisposing, precipitating, and perpetuating factors will allow progress toward understanding causal relations (including interactions and feedback) among changes in the identified networks, external factors, and the related dimensions of gender dysphoria, potentially discovering currently unseen doors for improving the lives of those with gender dysphoria.

## Synthesis

Reviewing Editor: Julie Bakker, University of Liege Decisions are customarily a result of the Reviewing Editor and the peer reviewers coming together and discussing their recommendations until a consensus is reached. When revisions are invited, a fact-based synthesis statement explaining their decision and outlining what is needed to prepare a revision will be listed below. The following reviewer(s) agreed to reveal their identity: Ivanka Savic, Nancy Forger.

I have received three reviews, one more negative and two more positive. However, I would advise to pay attention in particularly to reviewer 1 who states that your theory is not as new as it seems, and the omission of citing important papers already showing that gender dysphoria can be explained by changes in the network representing the perception of self.

Reviewer 1:

A new theory of gender dysphoria incorporating the distress, social behavioral,body-ownership, and sleep/wake networks.

The manuscript represents a ‘review’ of current literature supporting ‘authors new hypothesis’ that gender dysphoria is condition characterized by a disconnect involving one's sense of gender and gender roles, and altered sense of ownership of gendered body parts. In several ways, already from the very beginning the report reveals a surprising ignorance of the available literature the theory here presented as new, has both been formulated several years ago, thus, and, in addition, there are several publications showing supporting data, which the authors seem unaware aware of, or, omit to discuss.

Secondly, when discussing ‘social networks’ for gender behavior the authors seem to refer mainly to animal data, which inherently cannot be directly translatable to social gender behavior in humans. At least, the authors should indicate which statements are based only on animal data vs. not.

Third, the emphasis on the sleep wake cycle and its possible disturbance is a strech and poorly supported by the abundant clinical data on gender dysphoria. Consequently, the discussion about potential treatments via targeting the sleep wake cycle appears rather speculative.

Some details:

This It is somewhat remarkable that the published studies originally introducing this hypothesis, eg Manzouri et al.., 2017, 2018, Feusner&Savic were not cited, although each of these studies specifically introduce this hypothesis, and provide scientific data supporting it.

Raw 170, please provide reference to this statement

Raw 180, the statement is incorrect Kilpatrick et al., indeed reported effects of cross sex hormone treatment in relation to own body perception.

Comorbidity - why is Autism Spectrum Disorders not mentioned?

Reviewer 2:

This is a thoughtful and well-written paper presenting an intriguing new theory of gender dysphoria. The authors propose that in contrast to the “opposite sex brain” theory, gender dysphoria arises from altered functional activity in three networks - the stress/distress, body ownership, and social behavior networks - and name this the “gender-sense perception theory.”

I have several substantive concerns and a few minor comments/suggestions.

1) Lines 266 ff: “Under this alternate definition of brain sex, our results show that gender dysphoria is a functional, not anatomical, brain/body sex incongruence.” First, I suggest replacing the phrase “results show” with “hypothesis proposes.” Additionally, I wonder if you are setting up a false dichotomy? Network function depends on the number of projections, synapse number, synapse strength, etc... all of which are “anatomical.” It's true that the size of a brain area in and of itself doesn't “do” anything. But, implicit in size changes are changes in the number of cells or connections in a node. In other words, network function.

2) Lines 270 ff: “Rather, it appears that both females and males with gender dysphoria experience similar functional changes associated with the listed networks, thus supporting that gender dysphoria is not a variation in masculinity/femininity of the brain.” The main observation the proposed theory does not seem to account for is the opposite valence of the incongruence that transgender individuals experience: males who are transgender don't just feel disconnection with their bodies, but wish to be in a female body and females who are transgender wish to be in a male body. How does this arise, if the network activity changes are similar?

3) Lines 295ff: “The gender-sense theory is also consistent with two recent meta-analyses that found that brains of transgender individuals are actually distinct from brains of cisgender individuals of both genders (Guillamon et al., 2016; Smith et al., 2015).” The sentence does not really capture the conclusions of the papers cited. In Guillamon et al., male to female transsexuals were on average more feminine than males and female to male transsexuals were more masculine than females. Similarly, Smith et al. acknowledge some inconsistencies, but overall conclude “a selective feminization or masculinization of brain structures or processes that are sexually dimorphic in control subjects.”

4) Line 377ff: “However, anatomical brain sex only appears to be distinctive at the whole brain level, rather than at the level of individual nuclei, in cisgendered individuals (Chekroud et al., 2016; Joel et al., 2015; Rosenblatt, 2016).” I suggest removing the citation to Joel et al. (2015), because that paper actually says the opposite, if taken at face value. They find over 15 brain areas that are significantly different in size between males and females, but argue that there is no “female” or “male” brain overall. The other two citations do support the statement (in one case, using the Joel et al.'s data).

5) The paper is too long and some of the topics weaken the argument in my opinion. For example, the connection to the sleep/wake and circadian system is very tenuous and based on minimal anecdotal evidence. Since the overall theory is already speculative, this may be a “bridge too far.” I suggest deleting these portions of the paper as they appear in the Methods, Results and Discussion. (Related, the fact that the VMH has an endogenous clock does not really set it apart, as I believe most/many brain areas have now been shown to have endogenous clocks.) I also think that the case studies (page 14 and top of 15) should be deleted. It is possible to pick and choose cases to support almost any hypothesis and overall weakens the paper.

Minor comments/suggestions:

6) I assume that this is a Theory/New Concepts paper, as defined by eNeuro. The format of the paper seems a bit forced (methods, results) as it does not present any data. Is this the correct format?

7) Transgender versus transsexual. In some cases, papers are cited as showing something about “transgender” individuals when the original authors of those papers used the term “transsexual.” Some definition of terms may be warrented.

8) In several places throughout the manuscript, the word “effecting/effect” should be changed to “affecting/affect” (e.g., lines 253, 289, 293, 425).

Reviewer 3:

The author has proposed a new theory of gender dysphoria, as reflected in the title of the ms. In particular, the author advances a “gender-sense perception theory.”

In many respects, the paper appears thoughtful.

At the outset, I will be candid and state that I am not particularly qualified to evaluate the author's interpretation of the neuroimaging data and the analysis of brain function, etc. So, I will focus on other elements of the paper.

1. In my view, I would like the author to articulate much more clearly the role that sexual orientation plays in the theory. It is well-known that there are two subtypes of gender dysphoria in biological males: those who are sexually attracted to biological males and those who are sexually attracted to biological females (or those who are attracted to both biological males and females or who are “asexual”). Blanchard referred to these two subgroups as homosexual vs. non-homosexual. The author needs to read carefully Blanchard's typological work. One can also read Lawrence (2010, Arch Sex Behavior; 2017, European Psychologist). Regarding biological females, historically, the vast majority were sexually attracted to females although more recently we see more instances of those who are sexually attracted to males, so the homosexual vs. non-homosexual distinction can apply to biological females as well.

I bring this up early because on p. 2 the author refers to the Zhou et al. (1995) study and subsequent analysis of the sexual orientation of these deceased patients suggested that most of them, if not all of them, were “non-homosexual” (see Lawrence & Zucker, 2014, p. 671, Gender dysphoria. In D. C. Beidel, B. C. Frueh, and M. Hersen (Eds.), Adult psychopathology and diagnosis (Seventh ed.). Hoboken, NJ: John Wiley & Sons, 2014, pp. 603-639).

Regarding biological males, it is important to note that the homosexual subtype has a childhood history of marked gender-variant behavior whereas the non-homosexual subtype generally does not. So, what are the implications for the theory knowing that the latter subtype was “gender typical” during childhood, at least with regard to overt displays of gender expression?

On p. 6, Line 137, the author reports some structural MRI “controlling for sexual orientation”: the author needs to say what this actually means in terms of what was found.

On p. 12, Lines 279-280, the author seems to be making the case that sexual orientation is not that important in the model (I say this by inference, because age of onset is associated with the homosexual/non-homosexual distinction among biological males). The former are early-onset and the latter are late-onset.

On p. 13, Lines 295-298: Where does sexual orientation fit in with the summary of the meta-analyses?

2. P. 2, Line 41: It is not necessary to refer to Breedlove as “Dr. Breedlove.”

3. P. 3, Line 51: Is it premature to refer to the distress network without giving a citation?

4. P. 5, top para: Of course, many mental health conditions are associated with distress, so specificity seems to be an issue that I hope the author takes up later in the paper. I very much liked the proposed comparison conditions given at p. 18, Lines 404-405. BDD and anorexia would seem to be very good groups to study although it is interesting to note that these two conditions are much more common in females than in males.

5. P. 8, para 1: “Gender dysphoria is distinct from being gender-atypical...many gender-atypical individuals do not experience significant distress nor a decreased ownership of their assigned gender.” Agreed. So, propose what a comparison group of non-gender dysphoric gender-atypical individuals would tell us with regard to the key parameters in the new theory. Gay men with a childhood history of gender-variant behavior and lesbian women with a childhood history of gender-variant behavior would be good comparison groups, no?

6. P. 8, para 1: “...mediated by psychosocial factors.” Tell us what these psychosocial factors are.

7. P. 9, last sentence: “Behavior atypical of assigned gender is common in individuals with gender dysphoria...” But not in the non-homosexual males with gender dysphoria, at least during childhood. What are the implications of this for the theory?

8. P. 10, top para: “...anecdotal evidence suggests a higher incidence of sleep concerns in children with gender dysphoria.” This was news to me. I think the author has to be very cautious about this until there are more data. I think anecdotal is even too strong a statement. There is the well-known Child Behavior Checklist, which is a parent-report measure of behavioral and emotional problems in children and adolescents, with all items rated on a 0-2 point scale. There are, I think, 5 items on this questionnaire that might be relevant: “Trouble sleeping”; “Talks or walks in sleep”; “Sleeps more than most kids during day and/or night”; “Sleeps less than most kids”; “Overtired without good reason” (Items 54, 76, 77, 92, 100). It would be very interesting to do an item analysis and compare to referenced norms. The Amsterdam group probably has hundreds of CBCLs available on children and adolescents with gender dysphoria where the author could get this information. I think the Kern et al. citation on p. 13, Line 320 is insufficient.

9. P. 15, para 1: Here, what the author says is grossly simplistic. The Denny citation is hardly definitive. Aversion therapy to treat adults with gender dysphoria was almost never done (see the chapter by Marks and Gelder in Green and Money, 1969). And whatever was done by Marks and Gelder had nothing to do with gender atypical behavior. Now, in the 1970s, behavior therapists treating gender dysphoria in children using reinforcement paradigms, but these did not include aversion therapy techniques (Zucker, 1985 in Steiner, Gender dysphoria, Plenum Press summarized the behavior therapy treatment studies). I want to point out here that in very young children we don't see much in the way of “anatomical incongruence” (see Lambert, S. L. Assessment of body image in boys with gender identity disorder: A comparison to clinical control boys and community control boys. Doctoral dissertation, York University, 2009), so maybe this is one reason that we can't really predict very well which gender dysphoric children will persist or desist.

Minor points

1. Use the plural for data (data do, not data does; data challenge, not data challenges; data were, not data was; data have, not data has; data are, not data is; data question, not data questions).

2. Typo: gender identify to identity in several places; dysregulate, not disregulate

3. The two Steensma references are duplicates

## Author Response

- The species studied is not mentioned in the abstract. Please make sure to update both the abstract in the article file and on the submission form.

Response: the word “human” is now included in the abstract.

Computational Neuroscience Model Code Accessibility Comments for Author (Required):

N/A

Significance Statement Comments for Author (Required):

since it concerns a review paper and no real data paper, I would advise to avoid talking about “our results” in the significance statement.

Response: this has been done in the significance statement as well as throughout the manuscript.

Comments on the Visual Abstract for Author (Required):

N/A

Synthesis Statement for Author (Required):

I have received three reviews, one more negative and two more positive. However, I would advise to pay attention in particularly to reviewer 1 who states that your theory is not as new as it seems, and the omission of citing important papers already showing that gender dysphoria can be explained by changes in the network representing the perception of self.

Response: thank you. We have updated the manuscript to address all concerns. In particular, the manuscript now includes these important references and provides greater clarity regarding the novelty of the proposed theory. See below.

Reviewer 1:

A new theory of gender dysphoria incorporating the distress, social behavioral,body-ownership, and sleep/wake networks.

The manuscript represents a ‘review’ of current literature supporting ‘authors new hypothesis’ that gender dysphoria is condition characterized by a disconnect involving one's sense of gender and gender roles, and altered sense of ownership of gendered body parts. In several ways, already from the very beginning the report reveals a surprising ignorance of the available literature the theory here presented as new, has both been formulated several years ago, thus, and, in addition, there are several publications showing supporting data, which the authors seem unaware aware of, or, omit to discuss.

Response: thank you for bringing these important references to our attention. We have incorporated the several papers you cite below as well as others from the Savic group. We have revised the manuscript to clarify that 1) the connection between the body perception network and gender dysphoria is not new and is supported by a body of literature, and 2) the theory presented herein goes significantly beyond theories and ideas presented in the published literature, including papers by the Savic group. The references you provide strengthen a portion of our proposed theory. Specific changes to the manuscript include rewriting the paragraph describing changes found in the body ownership network to incorporate the work of Savic et al. and referencing the work of the Savic group in the introduction and in other relevant places.

Response continued: We also apologize for the lack of clarity in the manuscript that gave the wrong impression that our theory was already encompassed in the references you cite. Our theory is quite distinct and more broad than that from the group of Savic or elsewhere in the published literature. We have made modifications to the manuscript to make this distinction more obvious. In general, we have made minor adjustments to the text throughout to improve the clarity and specificity of the language. In particular, the distinctness between overall sense of gender and the contribution to this sense based on the body ownership network is now more clear. We also now clarify how our theory expands upon the work of Savic's group to also include aspects they do not, such as the distress and social behavioral networks as well as the integration of these three networks. For example, in the section presenting our theory, we have removed a paragraph about potential causal relations (moving the essence of the paragraph to the discussion) and instead include text and a figure explaining in greater detail the integration of information from the multiple involved networks (a key point demonstrating how our theory involves more than just the body-perception network). We have also changed the name of our theory from “gender-sense” to “multisense” to reinforce the relevance of multiple networks, not just one. We have also added new paragraphs to the “Comparison with other theories of gender dysphoria” section of the discussion which specifically clarifies how our theory extends beyond theories presented in two recent (2019) papers on gender dysphoria, including one with Savic as a senior author. Thus, the revised manuscript properly cites and recognizes the important work of the Savic group, including those papers you point out below, and also provides strong evidence how our proposed theory is new.

Secondly, when discussing ‘social networks’ for gender behavior the authors seem to refer mainly to animal data, which inherently cannot be directly translatable to social gender behavior in humans. At least, the authors should indicate which statements are based only on animal data vs. not.

Response: we have added text to clarify which statements are based on human vs. animal data as requested. We also directly acknowledge the limitation you raise, and provide references that provide more detail about applicability of the social behavioral network to humans.

Third, the emphasis on the sleep wake cycle and its possible disturbance is a strech and poorly supported by the abundant clinical data on gender dysphoria. Consequently, the discussion about potential treatments via targeting the sleep wake cycle appears rather speculative.

Response: based on your comment and those by other reviewers, we have now moved all mention of sleep/circadian to a short section in the discussion and removed sleep/circadian from the title. We also specifically removed the statement you reference. However, there is a lack of data regarding sleep in this population, and therefore we feel it important to at least discuss the possible relationship to help guide future research.

Some details:

This It is somewhat remarkable that the published studies originally introducing this hypothesis, eg Manzouri et al.., 2017, 2018, Feusner&Savic were not cited, although each of these studies specifically introduce this hypothesis, and provide scientific data supporting it.

Response: these studies are now cited, and the distinction between the hypothesis they test and the central hypothesis of this manuscript has been clarified in the manuscript. Their hypotheses specifically focused on the relevance of body ownership/perception, whereas our theory includes relationships between three networks and three dimensions of gender dysphoria, only one of which is the body ownership/perception network. Thank you for these important references.

Raw 170, please provide reference to this statement

Response: we have reworded the sentence to make it clear that we are not referring to specific empirical data (which should have a reference), but instead referring to general knowledge and definitions. We have also added a reference to the DSM-V, which recognizes that gender atypical behavior, without the presence of a certain level of distress, does not constitute gender dysphoria.

Raw 180, the statement is incorrect Kilpatrick et al., indeed reported effects of cross sex hormone treatment in relation to own body perception.

Response: thank you for bringing this paper to our attention, which strengthens several aspects of our manuscript. We now include a sentence addressing and citing the paper you mention.

Comorbidity - why is Autism Spectrum Disorders not mentioned?

Response: we now include autism in our list of comorbidities.

Reviewer 2:

This is a thoughtful and well-written paper presenting an intriguing new theory of gender dysphoria.

Response: thank you for your positive comments.

The authors propose that in contrast to the “opposite sex brain” theory, gender dysphoria arises from altered functional activity in three networks - the stress/distress, body ownership, and social behavior networks - and name this the “gender-sense perception theory.”

I have several substantive concerns and a few minor comments/suggestions.

1) Lines 266 ff: “Under this alternate definition of brain sex, our results show that gender dysphoria is a functional, not anatomical, brain/body sex incongruence.” First, I suggest replacing the phrase “results show” with “hypothesis proposes.”

Response: done. We have in fact replaced the word “results” when referring to aspects of this manuscript throughout the entire paper.

Additionally, I wonder if you are setting up a false dichotomy? Network function depends on the number of projections, synapse number, synapse strength, etc... all of which are “anatomical.” It's true that the size of a brain area in and of itself doesn't “do” anything. But, implicit in size changes are changes in the number of cells or connections in a node. In other words, network function.

Response: we apologize for the confusion. Rather than trying to clarify what we were trying to express, we note that this sentence is part of a paragraph discussing how the model might be understood under an alternate definition of brain sex. Given your later comment about the paper being too long and that some points weakening the argument, we have decided to remove this potentially confusing paragraph about a hypothetical alternate definition as it is not critical to the goals of the manuscript.

2) Lines 270 ff: “Rather, it appears that both females and males with gender dysphoria experience similar functional changes associated with the listed networks, thus supporting that gender dysphoria is not a variation in masculinity/femininity of the brain.” The main observation the proposed theory does not seem to account for is the opposite valence of the incongruence that transgender individuals experience: males who are transgender don't just feel disconnection with their bodies, but wish to be in a female body and females who are transgender wish to be in a male body. How does this arise, if the network activity changes are similar?

Response: this question refers to text within the paragraph removed for brevity (see response to your comment #1), though your question still applies to the overall theory. We have added text to the manuscript that specifically answers this question, as well as a citation supporting its relevance. The simple answer is that gender appears to be encoded in the brain as “same” vs “opposite” rather than “male” vs “female” (supported, in part, by Burke et al., 2019, “Sex differences in own and other body perception”). In terms of male and female, it seems the valence is opposite as you note. But in terms of “same” vs. “opposite” gender, the valence is the same: individuals of both sexes with gender dysphoria desire the body which is not the “same” as the one they have. Please see the text for further detail.

3) Lines 295ff: “The gender-sense theory is also consistent with two recent meta-analyses that found that brains of transgender individuals are actually distinct from brains of cisgender individuals of both genders (Guillamon et al., 2016; Smith et al., 2015).” The sentence does not really capture the conclusions of the papers cited. In Guillamon et al., male to female transsexuals were on average more feminine than males and female to male transsexuals were more masculine than females. Similarly, Smith et al. acknowledge some inconsistencies, but overall conclude “a selective feminization or masculinization of brain structures or processes that are sexually dimorphic in control subjects.”

Response: we apologize for the confusion and our lack of clarity between the data presented in these meta-analyses and their specific conclusion statements. We have updated our manuscript accordingly and now state: “...data presented show that brains of transgender individuals are not simply altered along a male/female dimension to be more like their desired gender.” While your statements and their conclusions are based on a qualitative average, I was clarifying that not all the data fits well with that average.

4) Line 377ff: “However, anatomical brain sex only appears to be distinctive at the whole brain level, rather than at the level of individual nuclei, in cisgendered individuals (Chekroud et al., 2016; Joel et al., 2015; Rosenblatt, 2016).” I suggest removing the citation to Joel et al. (2015), because that paper actually says the opposite, if taken at face value. They find over 15 brain areas that are significantly different in size between males and females, but argue that there is no “female” or “male” brain overall. The other two citations do support the statement (in one case, using the Joel et al.'s data).

Response: thank you. We have done as suggested.

5) The paper is too long and some of the topics weaken the argument in my opinion.

Response: thank you for bringing this to our attention. We have removed several sections that are less relevant or noted by reviewers to weaken the arguments, and have shortened other sections.

For example, the connection to the sleep/wake and circadian system is very tenuous and based on minimal anecdotal evidence. Since the overall theory is already speculative, this may be a “bridge too far.” I suggest deleting these portions of the paper as they appear in the Methods, Results and Discussion.

Response: we agree that the sleep/wake network is one of the weaker components given available published data. Based on your comment and those by other reviewers, we have now moved all mention of sleep/circadian to the discussion and removed it from the title. We did not remove it 100% from the paper, as we feel this is an important but understudied area and therefore worthy of mention. However, placing it in one small section of the discussion allows us to acknowledge its weakness without overly weakening the main goals and flow of the full manuscript.

(Related, the fact that the VMH has an endogenous clock does not really set it apart, as I believe most/many brain areas have now been shown to have endogenous clocks.)

Response: this statements was removed when moving the sleep/circadian from the main body of the paper.

I also think that the case studies (page 14 and top of 15) should be deleted. It is possible to pick and choose cases to support almost any hypothesis and overall weakens the paper.

Response: we have done as you recommended and have removed the case studies.

Minor comments/suggestions:

6) I assume that this is a Theory/New Concepts paper, as defined by eNeuro. The format of the paper seems a bit forced (methods, results) as it does not present any data. Is this the correct format?

Response: yes, it is a “Theory/New Concepts” paper. We agree that the format does seem forced, but the online guide for authors stated such format was required with no stipulation for Theory/New Concept papers. I have contacted the reviewing editor and was informed that I am allowed to deviate from the prescribed methods, results, etc. format. The manuscript has now been updated to use more appropriate formatting and section labels. The order of a few of the paragraphs in the discussion has also been adjusted to allow for better flow and organization.

7) Transgender versus transsexual. In some cases, papers are cited as showing something about “transgender” individuals when the original authors of those papers used the term “transsexual.” Some definition of terms may be warrented.

Response: we have included the following statement addressing transgender vs. transsexual in the introduction as requested: “We also use the term ‘transgender’ throughout this manuscript, though recognize that some references instead use the word transsexual to refer to the same concept.”

8) In several places throughout the manuscript, the word “effecting/effect” should be changed to “affecting/affect” (e.g., lines 253, 289, 293, 425).

Response: thank you. Each instance was reviewed and corrected.

Reviewer 3:

The author has proposed a new theory of gender dysphoria, as reflected in the title of the ms. In particular, the author advances a “gender-sense perception theory.”

In many respects, the paper appears thoughtful.

At the outset, I will be candid and state that I am not particularly qualified to evaluate the author's interpretation of the neuroimaging data and the analysis of brain function, etc. So, I will focus on other elements of the paper.

1. In my view, I would like the author to articulate much more clearly the role that sexual orientation plays in the theory. It is well-known that there are two subtypes of gender dysphoria in biological males: those who are sexually attracted to biological males and those who are sexually attracted to biological females (or those who are attracted to both biological males and females or who are “asexual”). Blanchard referred to these two subgroups as homosexual vs. non-homosexual. The author needs to read carefully Blanchard's typological work. One can also read Lawrence (2010, Arch Sex Behavior; 2017, European Psychologist). Regarding biological females, historically, the vast majority were sexually attracted to females although more recently we see more instances of those who are sexually attracted to males, so the homosexual vs. non-homosexual distinction can apply to biological females as well.

I bring this up early because on p. 2 the author refers to the Zhou et al. (1995) study and subsequent analysis of the sexual orientation of these deceased patients suggested that most of them, if not all of them, were “non-homosexual” (see Lawrence & Zucker, 2014, p. 671, Gender dysphoria. In D. C. Beidel, B. C. Frueh, and M. Hersen (Eds.), Adult psychopathology and diagnosis (Seventh ed.). Hoboken, NJ: John Wiley & Sons, 2014, pp. 603-639).

Response: thank you for bringing up this important point. We have added a section to the discussion to address these questions, entitled “Interaction with other networks: sexual and romantic partner preference.” We did not include sexual attraction in the main body of the paper (or main theory) as we felt the neurobiological data on sexual partner preference in humans is not yet sufficiently strong.

Regarding biological males, it is important to note that the homosexual subtype has a childhood history of marked gender-variant behavior whereas the non-homosexual subtype generally does not. So, what are the implications for the theory knowing that the latter subtype was “gender typical” during childhood, at least with regard to overt displays of gender expression?

Response: that is an interesting question and highlights the dynamic aspect of this theory. Your note about play and the subtypes is consistent with the multisense theory, as the theory allows variability in the timing and order of when each of the networks are affected. It also allows feedback with external stimuli. For example, gender variant childhood play could result in negative external feedback, causing distress, and exacerbating changes in the distress network. Thus the negative external feedback (not the gender variant play) may be a precipitating factor to early onset gender dysphoria. Unfortunately, we do not know enough at present, and thus it is too speculative to directly address this question in the text.

On p. 6, Line 137, the author reports some structural MRI “controlling for sexual orientation”: the author needs to say what this actually means in terms of what was found.

Response: the specific text was changed when incorporating the additional references from Reviewer #1. However, we have still sought to clarify this point when the concept of “controlling for sexual orientation” is mentioned.

On p. 12, Lines 279-280, the author seems to be making the case that sexual orientation is not that important in the model (I say this by inference, because age of onset is associated with the homosexual/non-homosexual distinction among biological males). The former are early-onset and the latter are late-onset.

Response: the new section “Interaction with other networks: sexual and romantic partner preference” discusses the relevance of sexual orientation in our theory. We specifically include a paragraph detailing how our theories can describe the observed relationship between onset age and the homosexual/non-homosexual distinction among biological males. Also please note, recent data questions association with early-onset and sexual orientation. In Zavlin et al., (2019), the authors concluded that the distribution of subtypes is statistically different between early (<18 years old) and late onset cases. However, their data also show that the amount of homosexual vs. non-homosexual subtypes was almost 50-50 in early onset cases.

On p. 13, Lines 295-298: Where does sexual orientation fit in with the summary of the meta-analyses?

Response: we have reworded this section to improve clarity and added the phrase “even in studies which controlled for sexual orientation” to answer this question.

2. P. 2, Line 41: It is not necessary to refer to Breedlove as “Dr. Breedlove.”

Response: thank you. We have now corrected this.

3. P. 3, Line 51: Is it premature to refer to the distress network without giving a citation?

Response: we have added a citation.

4. P. 5, top para: Of course, many mental health conditions are associated with distress, so specificity seems to be an issue that I hope the author takes up later in the paper. I very much liked the proposed comparison conditions given at p. 18, Lines 404-405. BDD and anorexia would seem to be very good groups to study although it is interesting to note that these two conditions are much more common in females than in males.

Response: thank you for your positive comment.

5. P. 8, para 1: “Gender dysphoria is distinct from being gender-atypical...many gender-atypical individuals do not experience significant distress nor a decreased ownership of their assigned gender.” Agreed. So, propose what a comparison group of non-gender dysphoric gender-atypical individuals would tell us with regard to the key parameters in the new theory. Gay men with a childhood history of gender-variant behavior and lesbian women with a childhood history of gender-variant behavior would be good comparison groups, no?

Response: discussion of alternate control groups are proposed in the Discussion section, “Future directions.” Individuals with gender-variant behavior were already listed, but we now include the phrase “of each sexual orientation” and we specify the atypical behavior may be “during childhood or other ages”. We also describe how the extra control groups will help disambiguate the relative impact of each brain region to each dimension of gender dysphoria.

6. P. 8, para 1: “...mediated by psychosocial factors.” Tell us what these psychosocial factors are.

Response: we removed this phase, as detailing this is beyond the scope of this paper and is not directly relevant.

7. P. 9, last sentence: “Behavior atypical of assigned gender is common in individuals with gender dysphoria...” But not in the non-homosexual males with gender dysphoria, at least during childhood. What are the implications of this for the theory?

Response: we have added the phrase “(with some exceptions depending on age of onset and sexual orientation).” The further implications for the theory are the potential interaction between different networks, which we now discuss in the “Interaction with other networks: sexual and romantic partner preference” section. See also earlier answer (part of response to question set 1) regarding similar question.

8. P. 10, top para: “...anecdotal evidence suggests a higher incidence of sleep concerns in children with gender dysphoria.” This was news to me. I think the author has to be very cautious about this until there are more data. I think anecdotal is even too strong a statement.

Response: based on your comment, we have weakened the statement. We have changed the wording to “We do note that one case study makes an unsupported statement that sleep disorders are higher in children with gender dysphoria (Kern et al., 2014), though direct empirical evidence does not seem to be available.”

There is the well-known Child Behavior Checklist, which is a parent-report measure of behavioral and emotional problems in children and adolescents, with all items rated on a 0-2 point scale. There are, I think, 5 items on this questionnaire that might be relevant: “Trouble sleeping”; “Talks or walks in sleep”; “Sleeps more than most kids during day and/or night”; “Sleeps less than most kids”; “Overtired without good reason” (Items 54, 76, 77, 92, 100). It would be very interesting to do an item analysis and compare to referenced norms. The Amsterdam group probably has hundreds of CBCLs available on children and adolescents with gender dysphoria where the author could get this information. I think the Kern et al. citation on p. 13, Line 320 is insufficient.

Response: these are helpful suggestions for future work, but beyond the scope of this manuscript. To help support such future work, we feel it is important to at least mention the possible connection between sleep/circadian and gender dysphoria in the discussion.

9. P. 15, para 1: Here, what the author says is grossly simplistic. The Denny citation is hardly definitive. Aversion therapy to treat adults with gender dysphoria was almost never done (see the chapter by Marks and Gelder in Green and Money, 1969). And whatever was done by Marks and Gelder had nothing to do with gender atypical behavior. Now, in the 1970s, behavior therapists treating gender dysphoria in children using reinforcement paradigms, but these did not include aversion therapy techniques (Zucker, 1985 in Steiner, Gender dysphoria, Plenum Press summarized the behavior therapy treatment studies). I want to point out here that in very young children we don't see much in the way of “anatomical incongruence” (see Lambert, S. L. Assessment of body image in boys with gender identity disorder: A comparison to clinical control boys and community control boys. Doctoral dissertation, York University, 2009), so maybe this is one reason that we can't really predict very well which gender dysphoric children will persist or desist.

Response: given your concerns with this section and Reviewer #2's comments that “The paper is too long and some of the topics weaken the argument in my opinion,” we have removed the referenced paragraph. The first theory we consider in the comparison with other theories is now the opposite brain sex theory.

Minor points

1. Use the plural for data (data do, not data does; data challenge, not data challenges; data were, not data was; data have, not data has; data are, not data is; data question, not data questions).

2. Typo: gender identify to identity in several places; dysregulate, not disregulate

3. The two Steensma references are duplicates

Response: thank you for noting these. All have been corrected as you suggest.
